The article "Development of a Sandwich Enzyme-Linked Immunosorbent Assay for Detection and Quantification of Clam Residues in Food Products" was published in 2021. Journal: Biomed Res Int.

# Development of a Sandwich Enzyme-Linked Immunosorbent Assay for Detection and Quantification of Clam Residues in Food Products

**DOI:** 10.1155/2021/6685575

**Published:** 2021-03-19

**Authors:** Stef J. Koppelman, Ashley L. Lardizabal, Lynn Niemann, Joe L. Baumert, Steve L. Taylor

**Affiliations:** Food Allergy Research and Resource Program, Department of Food Science and Technology, University of Nebraska, Lincoln, NE 68583-0955, USA

## Abstract

Seafood is a frequent cause of allergic reactions to food globally. The presence of undeclared trace amounts of clam can cause allergic reactions in sensitive individuals. Limited tools are available to test food products for the presence of traces of clam. We report on the development of a sandwich ELISA that can detect and quantify clam protein in food. Antisera against a mix of two commercially important clam species, Atlantic Surf (*Spisula solidissima*) and ocean quahog (*Arctica islandica*), were raised in rabbit and sheep. A sandwich ELISA was constructed with this antisera, and sensitivity and specificity were evaluated. Also, model food products spiked with clam protein were analyzed to assess the performance of the ELISA. Comparison was made with a commercially available ELISA for crustacea. The lower limit of quantification of the sandwich ELISA is 2.5 ppm clam protein in food samples, allowing the detection of low amounts of clam that may trigger a reaction in clam allergic patients. The sandwich ELISA was highly specific with cross-reactivity only noted for other molluscan shellfish (mussel and scallop). Clam protein in tomato juice and potato cream soup was detected well with recoveries ranging from 65 to 74% and from 74 to 113%, respectively. However when potato cream soup was retorted, the recover fell to 20%, imposing the risk of underestimating the clam content of a food product. A commercially available crustacean ELISA test was not suitable to detect clam protein. The sandwich ELISA described here is suitable for detection and quantification of clam protein in food products. Care should be taken with food products that have been retorted as the results may be underestimated.

## 1. Introduction

Clams are molluscan shellfish, part of the second largest phylum in the animal kingdom having 104 edible species according to the Food & Agriculture Organization of the United Nations. Molluscan shellfish are sometimes grouped together with crustacean shellfish (shrimp, crab, lobster, etc.) but, in fact, molluscan and crustacean shellfish belong to two quite distinct phyla. Molluscan shellfish are further subdivided into 9-10 classes with three classes that are commonly ingested—bivalves (clams, oysters, mussels, scallops, etc.), cephalopods (squid, octopus, and cuttlefish), and gastropods (snails, abalone, limpet, etc.). Clams belong to the *Bivalvia* (bivalves) class of the *Mollusca* phylum. While there are many species of clam, the ocean quahog and Atlantic Surf clam are the primary species used commercially in the US. In the US, the production of ocean quahog clams was 11.3 million pounds in 2019, while the production of Atlantic Surf clams was 37 million pounds in 2017 (http://www.fishwatch.gov).

Commercially, the vast majority of clam meat produced is used for canned products such as whole, minced, chowder, juice, and specialty products. Atlantic Surf clam (*Spisula solidissima*) is one of the largest species inhabiting the Atlantic coast with a typical shell length of 7 to 8 inches. The Atlantic Surf clam is also known as skimmer, hen clam, sea clam, or bar clam. These clams are not sold live or whole. Market forms of surf clams include chopped, frozen, individually quick frozen (IQF), or canned including prefried strips, breaded, chowders, bisques, and clam juice (http://www.fishwatch.gov). The surf clam is the only clam that is used in manufacturing frozen, breaded clam strips. The shucked meat of the surf clam includes the “tongue” which is often used to make fried clam strips and the strap meat which is ground or chopped and used for chowders, bisques, and sauces. The ocean quahog (*Arctica islandica*) is somewhat smaller (2.8 to 4.3 inches in shell length) and is marketed for in-shell preparation as well. This clam is known by a variety of names including mahogany clam, mahogany quahog, ocean clam, or black clam. Ocean quahog meat is strongly flavored and is often used in products that are complemented by this taste, such as tomato-based recipes. These clams are generally minced, chopped, or cut into strips before they are suitable for the table. The Northern quahog or hard clam (*Mercenaria mercenaria*) is another commercial species in the US but annual production of Northern quahog is substantially lower than that of ocean quahog and Atlantic Surf clam (http://www.fishwatch.gov).

Both molluscan and crustacean shellfish are well-known causes of IgE-mediated, immediate hypersensitivity allergic reactions [1, 2]. Crustacean shellfish allergies are perhaps the most prevalent food allergy globally with estimates from self-report surveys in the US as high as 2% [3–6]. When clinical confirmation is sought, the prevalence rate drops to less than half of these estimates [7]. The prevalence of molluscan shellfish allergy has not been thoroughly assessed. Self-report surveys in the US indicated that the prevalence of molluscan shellfish allergy is between 0.4% and 0.5% [5, 6]. A questionnaire-based survey of 2716 school children in France estimated that the prevalence of molluscan shellfish allergy was 0.15% [8]. However, none of the allergies reported in France involved clams. In a survey of patients with food allergies from 17 clinics in 15 cities in the Baltic region of the EU, 6.2% of the participants indicated an allergy to clams [9]. However, clinical confirmation of these survey responses was not conducted. In several studies of food-allergic patients at separate clinics in Spain, 10/355 (2.8%) and 10/120 (8.3%), respectively, reported allergies to clams without further clinical confirmation [10, 11]. Skin testing of 625 Japanese asthmatic adults showed that 6.9% were sensitized to a clam extract but again food challenges were not conducted to confirm reactivity to clam [12]. In a nationwide survey of 30,018 individuals in Taiwan, 1.2% reported allergies to molluscan shellfish [13] but clinical confirmation was not sought.

The clinical literature contains very few well-documented case reports of IgE-mediated clam allergy. Clam allergy was first reported as early as 1916 [14, 15]. Parker et al. [16] described two clam allergic patients; one had gastrointestinal symptoms on oral challenge while the other had a history of laryngeal edema and was not challenged. Jiménez et al. [17] described an adult woman who experienced pruritis and facial angioedema on three occasions after eating razor clams. In addition, clams have been implicated in several cases of food protein-induced enterocolitis syndrome or FPIES [18, 19].

Individuals with shellfish allergies (either molluscan or crustacean or both) often avoid consumption of all shellfish species. Considerable biological diversity occurs within the molluscan phylum, and even more diversity exists between the molluscan and crustacean phyla so the likelihood of cross-reactivity among the many species within the molluscan phylum or across the molluscan and crustacean phyla seems unlikely, although some individuals do have cross-sensitivity to both molluscan and crustacean species [2]. The muscle protein, tropomyosin, seems to be a major allergenic protein in both molluscan and crustacean species [20, 21] but sequence homology between molluscan and crustacean species is sufficiently different that cross-reactivity is not common [2, 22]. The allergens in clam have not been widely studied but tropomyosin is identified as an allergen in four clam species: short-neck clam (*Ruditapes philippinarum*), Sakhalin surf clam (*Spisula sachalinensis*), razor clam (*Solen strictus*), and horse clam (*Tresus keenae*) [20]. Furthermore, cross-reactivity within the bivalve class has not been clinically investigated.

Avoidance of clam ingestion is the main preventive measure taken by clam-allergic consumers. Because of the use of shared processing facilities and equipment in the food industry, a risk exists of cross contact of clam with other food products occurring in certain situations. Cross contact can lead to unintended allergen presence in other food products which could pose a risk to clam-allergic consumers. The proper labeling of packaged foods is critical to the implementation of a successful clam avoidance diet. Therefore, reliable detection and quantification methods for food allergens are needed in order to guarantee compliance with food labeling regulations, to validate the effectiveness of allergen control measures in shared use facilities, and to improve consumer protection. Enzyme-linked immunosorbent assay (ELISA) is currently successfully used for analysis of other food allergens like milk, egg, walnut, and peanut [23–27]. We report the development of a sensitive and specific ELISA for the detection of clam residues in foods, based on the use of polyclonal antisera raised against a mixture of processed clam proteins.

## 2. Materials and Methods

### 2.1. Immunogen Preparation

Ocean quahog (*Arctica islandica*) and Atlantic Surf clam (*Spisula solidissima*) were used for the immunogen preparation. Clams were purchased from J. H. Miles Seafood Company (VA) and Blount Seafood Company (MA). The raw, thawed, and chopped clam meat obtained from the suppliers was thoroughly washed 3 times with distilled water. The meats were ground separately using a commercial food processor (KPF600 Food Processor, Kitchen Aid®, St. Joseph, MO). The cooked clams were prepared by mixing raw clam meat from each species in a 1 : 5 (w/v) ratio in deionized water and boiling for 3-5 minutes. Equal portions of each clam species were mixed, packed in hermetically sealed containers in water, and thermally processed in a static retort for 70 minutes at 250°F and 15 psi. Using the Kjeldahl method, the crude protein of this processed clam was determined and diluted with water to obtain a 2 mg/mL concentration of protein for use as the immunogen.

### 2.2. Polyclonal Antibody Production and Titer Determination

Polyclonal antibodies were produced at Covance Research Products (Denver, PA). The processed clam immunogen was used to immunize three New Zealand white rabbits and one sheep. The processed clam protein was emulsified with Complete Freund's Adjuvant (CFA) and administered to the rabbits intradermally and to the sheep subcutaneously. Every 21 days thereafter, booster injections were applied subcutaneously with the protein emulsified with Incomplete Freund's Adjuvant (IFA). Two weeks after each booster injection, a serum sample was collected for titer testing. Titer values of collected antisera were determined by a noncompetitive ELISA method in which log dilutions of serum were applied to plates coated with 1 *μ*g of processed clam protein per well in a coating buffer (15 mM Na_2_CO_3_, 35 mM NaHCO_3_, and 0.02% NaN_3_, pH 9.6) at 100 *μ*L per well, as previously described [24]. The titer values of the antisera were calculated using the Prism Windows-based computer software (GraphPad Software Inc., San Diego, CA) to determine the dilution of antibody at the midpoint of the linear portion of the dilution curve. Sera with titers of 10,000 and higher were kept and pooled per species. Titers performed on sera obtained from animals prior to immunization indicated that none of the animals possessed preexisting antibodies to clam.

Polyclonal antibodies were partially purified from the sera by precipitation with ammonium sulfate [28]. The partially purified IgG was dialyzed against deionized water and then extensively dialyzed against 10 mM phosphate buffered saline (PBS; 2 mM NaH_2_PO_4_, 8 mM Na_2_HPO_4_, 0.85% NaCl, and 0.02% NaN_3_, pH = 7.4) [23]. The dialyzed antibodies were then aliquoted and stored frozen at -20°C.

### 2.3. Clam Standards

The protein content of the processed/canned clam immunogen extracts prepared as described earlier was determined by the Lowry method [29]. Standard clam solutions were prepared using the clam immunogen extracts diluted in PBS at different levels of clam protein (1,000, 500, 250, 100, 50, 25, 12.5, 6.25, 3.125, 1.56, 0.78, and 0 ppm, with ppm being parts of clam protein per million parts of unextracted food sample).

### 2.4. Sandwich ELISA for Clam

96-well microtiter plates (Maxisorp, Nalge Nunc International, Rochester, NY) were coated with 100 *μ*L and 3 *μ*g/mL sheep anti-processed clam antibody protein in coating buffer (15 mM Na_2_CO_3_, 35 mM NaHCO_3_, and 0.02% NaN_3_, pH 9.6). Coated microtiter plates were incubated overnight at 4°C and then washed four times with PBS-T (PBS containing 0.05% Tween 20 (BioRad Laboratories, Inc., Hercules, CA) in 10 mM PBS and 0.02% NaN_3_, pH 7.4) using a programmable automatic plate washer (AM60, DynesTechnologies, Inc., Chantilly, VA). Unused binding sites were blocked using 350 *μ*L per well of 0.1% gelatin (300 bloom porcine [Sigma-Aldrich Company, St. Louis, MO] in 0.1 M PBS, pH 7.4) followed by incubation for 1 hour at 37°C. Excess blocking agent was removed by washing 4 times with PBS-T. Then, 100 *μ*L of each standard or sample extract was applied to wells in triplicate, and plates were incubated for 1 hour at 37°C. After washing 4 times with PBS-T, bound clam protein was incubated with 2.0 *μ*g/mL of rabbit anti-processed clam antibody protein (detection antibody; 100 *μ*L and 10 mM PBS containing 0.1% Bovine Serum Albumin (Fraction V USB Corporation, Inc., Cleveland, Ohio)). After washing 4 times with PBS-T, the bound detection antibody was stained by successive addition to each well of 100 *μ*L of commercial goat anti-rabbit immunoglobulin G labeled with alkaline phosphatase (Pierce Biotechnology, Inc. Rockford, IL) diluted 1 : 5,000 in 10 mM PBS-BSA, pH 7.4 with incubation at 37°C for 1 hour, washing 4 times with PBS-T, and 100 *μ*L of *p*-nitrophenyl phosphate substrate (Sigma-Aldrich Company, St. Louis, MO) with incubation for 30 minutes at 37°C. Color development was read on a microplate reader (ELx808 Ultraplate Reader, Bio-Tek Instruments, Inc., Chantilly, VA) at 405 nm after stopping the reaction by addition of 100 *μ*L of 1 N sodium hydroxide to each well. The calibrant for the standard curve was an extract of the processed clam meat described earlier with results expressed as parts per million soluble clam protein. Standard curves were prepared using the Prism Windows-based computer software (GraphPad Software Inc., San Diego, CA) and were based on triplicate readings for each data point. Results are expressed as parts per million (ppm) in the unextracted sample (i.e., the dilution factor and extraction ratio have been taken into account).

### 2.5. Commercial ELISA for Crustacean

A commercially available ELISA kit specific for the detection of tropomyosin in crustacean shellfish (ELISA Systems Crustacean Residue ELISA; Windsor Queensland, Australia) was evaluated for its ability to detect and quantify various shellfish species. The foods tested were raw and cooked shrimp, lobster, crab, and clams. The assay was performed according to the manufacturer's instructions. Results are expressed as parts per million tropomyosin.

### 2.6. Food Samples and Extraction

A total of ninety-five foods/food ingredients were evaluated for cross-reactivity in the ELISA. Food samples were purchased from local grocery and specialty stores in Lincoln, NE. Solid samples were ground to uniform consistency using an Osterizer® blender (Sunbeam Corporation, Delray Beach, FL) or a commercial food processor (KPF600 Food Processor, Kitchen Aid®, St. Joseph, MO). Liquid and oil samples were used as is, and the diagnostic extracts were diluted in the assay.

Samples were extracted 1 : 10 (w/v) in 0.01 M PBS using gentle shaking (Labquake™ Shaker, Barnstead-Thermolyne Corporation, Dubuque, IA), overnight at room temperature. Guar gum was extracted at a 1 : 100 (w/v) ratio due to the gelling at higher w/v ratios. Samples were centrifuged at 4,066 x g (5,000 rpm) for 30 minutes at 4°C in a Sorvall® RC 5B Plus model centrifuge (Kendro Laboratory Products, Newton, CT), and the aqueous supernatants were stored at -20°C for later use. Oil samples were extracted 1 : 5 (w/v) in 0.01 M PBS at 140 rpm in a shaking water bath (JulaboSW22, Julabo USA, Inc., Allentown, PA) at 60°C for 2 hours. In some cases, the aqueous extract was concentrated using Centriprep® YM-3 concentrator (3,000 molecular weight cut-off, Amicon® Bioseparations, Millipore Corporation, Bedford, MA) following the manufacturer's instructions. Extraction ratios and concentration factors were taken into account when calculating the results. The protein content of extracts was determined using the Lowry method [29].

For cross-reactivity studies, extracts were tested in the sandwich ELISA undiluted, 10-fold, 100-fold, and 1,000-fold diluted. Positive samples were further diluted and retested. Dilutions giving responses in the sensitive range of the ELISA were used for calculations. Results are presented at W/W percentage of clam reactivity: (*clam reactivity* (*μg/mL*) *as measured with ELISA*) divided by (*protein concentration of the extract* (*μg/mL*)) multiplied by 100%.

### 2.7. Model Food Products

Tomato juice was obtained from a local grocery store in Lincoln, NE, and the ready-to-eat cream of potato soup was obtained from a local food distributor in Lincoln, NE. Both products were spiked directly with the appropriate amounts of nonprocessed clam extract at 0, 5, 10, 25, 50, and 100 ppm of clam protein. Spiked products were mixed thoroughly using a commercial mixer ((Legacy™ HL200) Mixer, Hobart Corporation, Troy, OH), resulting in six concentrations each of clam spiked into tomato juice and cream of potato soup. A portion of each of the cream of potato soup model food products was retorted in 12 oz commercial jars for 70 minutes at 245°F (118.3°C) in a static retort (Dixie Canner Equipment Co., Athens, GA).

## 3. Results and Discussion

### 3.1. Characterization of the Antisera

The reactivity of the sera for clam proteins was tested using IgG immunoblotting.  Figure 1(a) shows the protein patterns of native and processed Atlantic Surf and ocean quahog clams, and Figures 1(b) and 1(c) show the reactivity of the rabbit and sheep antibodies against these proteins.

For the raw samples, distinct protein bands can be observed at approximately 40 and 50 kDa, as well as at some other MWs both in the lower and higher range. These bands are also visible in the cooked samples. However, processing by retorting leads to a smear of protein stain without distinct bands (Figure 1(a)). The antibodies are raised against processed clam protein of both species and are reactive to native and cooked clam of both species (Figures 1(b) and 1(c)), but the two distinct bands at approximately 40 and 50 kDa observed in the protein profile are not the most dominant bands in the immunoblot. Presumably, the clam proteins were denatured upon processing and induced antibodies against the denatured structures that are only partially reactive to native clam protein. Because allergens have not been identified from these clam species, the capability of the sheep and rabbit antibodies to recognize clam allergens is unknown. The presence of detectable clam protein likely indicates the presence of clam allergens especially since whole clam meat is used in most food formulations.

### 3.2. Sandwich ELISA for Clam Protein: Sensitivity

Initial sandwich ELISA tests showed that optimal results were obtained using sheep anti-clam antibody, at a protein concentration of 3.0 *μ*g/mL, as the primary capture antibody and rabbit anti-clam antibody, at a protein concentration of 2.0 *μ*g/mL, as the detector antibody. The protein content for the processed clam extract was 2.55 mg/mL. The calibration curve for the processed clam extract (Figure 2) shows a dynamic range for the ELISA of 0.78 to 1,000 ppm of clam protein (relative to unextracted food sample weight) with a lower limit of quantification (LLOQ, defined as the concentration giving an absorbance of at least two times the background) of 2.5 ppm.

The ELISA was not evaluated for its sensitivity in detecting raw clam protein because clams are typically heat-processed in food formulations. The minimal eliciting or threshold dose for clam protein in clam-allergic individuals is not known but such threshold doses are known for several other allergenic foods and were related to analytical methods to quantify allergens in food [30]. Based on the mean dose for 10 food allergens needed to provoke an objective allergic reaction in the 1% most sensitive segment of the food-allergic population [30] and using a conservatively high consumption amount of 250 g of whole clam, the mean action level for analytical methods should be 7 ppm. Using this figure as a proxy, our ELISA is likely sufficiently sensitive to protect clam-allergic consumers from undeclared clam residues.

### 3.3. Sandwich ELISA for Clam Protein: Specificity

The sandwich clam ELISA was highly specific for the detection of clam protein residues (Table 1). The majority of the tested food and food ingredients derived from plants and animals (excluding seafood) that were not cross-reactive (<0.02% reactivity compared to clam). The only exception was ginger extract that gave a minor cross-reaction (0.02% compared to clam, a level which is very close to the cut-off).

When cross-reactivity was assessed with seafood (Table 2), a higher probability for cross-reactivity existed with other molluscs and crustaceans due to their closer phylogenetic relation with clam. A quantifiable but minor reactivity was found for crab and abalone (<0.1% compared to clam). Scallop and mussels show some cross-reactivity (0.23% and 1.4% compared to clam, respectively), most likely due to homologies in protein within the molluscs phylum. Tropomyosin is a well-studied protein across many species. The sequence of clam tropomyosin for homology searches with the Internet-based program BLAST (http://www.uniprot.org, accession code G8XWU1) showed 74-76% homology with abalone species, 68-72% homology with scallop species, and 66-68% homology with mussel species. Tropomyosin from crustacean species (lobster, crab, shrimp, and prawn) had all lower degrees of homology with clam (<58%).

Other proteins from the mollusc family are not so well documented and could not be used to determine homologies. Such proteins could play a role as well in determining the ELISA cross-reactivity because tropomyosin represents only a minor part of the total protein content of molluscs. The weak reactivity of these foods is unlikely to be noticed when they are present in lower amounts in typical food formulations.

Surimi made from pollock tested weakly positive in the sandwich ELISA for clam, while pollock itself did not (Table 2). Surimi may be flavored with fractions of cooking water used in the manufacture of canned shellfish, such as clams and scallops [31, 32]. Thus, trace amounts of clam protein may be present in the flavoring extract applied to the surimi during manufacturing.

### 3.4. Detection and Quantification of Clam Protein in Model Food Products Using the Sandwich ELISA

The capability of the sandwich ELISA to detect and quantify clam protein residues was assessed in several model foods—tomato juice and cream of potato soup (both unprocessed and retorted)—spiked with clam extract at 0, 5, 10, 25, 50, and 100 ppm protein.  Table 3 shows the recovery of clam protein in the different food products.

The lowest spike of 5 ppm clam protein could not be detected, probably because this value is very close to the LLOQ of the ELISA (2.5 ppm clam protein, see above). In tomato juice and cream of potato soup, the spikes of 10 to 100 ppm of clam protein could be detected and quantified. The recovery of clam protein from tomato juice was 65-74%, and in the case of cream of potato soup, recovery was 74-113%. Such recoveries are considered reasonable as ELISA ideally has recoveries in the range of 80–120% [33]. For retorted cream of potato soup, however, the spikes with 10 and 25 ppm clam protein could not be detected. The spikes of 50 and 100 ppm clam protein had low recoveries of about 20% (Table 3). This low recovery represents a risk for false negative test results with retorted food products. The high-heat treatment involved in canning/retorting could possibly be affecting the solubility of the protein or it could also be changing the antigenic properties of the clam proteins [34] limiting their detection with this ELISA. Since the antisera were raised against retorted clam extract, structural changes in the antigen(s) seem a less plausible explanation.

### 3.5. Detection of Clam Protein by Other Methods

Several other methods have been developed for the detection of molluscan shellfish residues [35–37]. Unterberger et al. [36] developed a multiplex ligation-dependent probe amplification method for the simultaneous detection of fish, cephalopods, and bivalves. This DNA probe had a reported sensitivity of 20 ppm for fish and bivalve residues and 100 ppm for cephalopod residues. The bivalve-specific probe was not actually tested against clam species and failed to work properly for the detection of scallop residues necessitating the addition of a specific scallop DNA probe to this multiplex method [36]. Sathe and Sharma [34] developed a multiplex polymerase chain reaction (PCR) method with capillary electrophoresis for the detection of tropomyosins from oyster, mussel, abalone (a gastropod species), and clam. The species of clam was the short-neck clam (*Ruditapes philippinarum*) commonly consumed in Southeast Asia. This method was not evaluated for its capability to detect residues of North American clams, ocean quahog, and Atlantic Surf clam. A commercial PCR method for the detection of mollusc residues is available from r-Biopharm in Germany. The capability of this method to detect the primary North American clam species has not been evaluated to our knowledge. PCR methods detect DNA residues for the allergenic food and can be highly specific if a very specific DNA primer is used. Since allergens are proteins, PCR and other DNA detection methods offer indirect proof of the presence of allergen residues. Protein and DNA residues may not always have the same fate in food processing operations. The detection of protein residues through use of ELISA methods offers a more direct indication of the presence of allergen residues. Zhang et al. [37] developed a sandwich ELISA method for the detection of tropomyosin from molluscan bivalves (clam, scallop, and cockle). This method uses a monoclonal antibody directed against a C-terminal peptide of tropomyosin that serves as an IgE-binding epitope [37]. This sequence of this C-terminal peptide is conserved across crustacean and molluscan species [20]. Zhang et al. [37] demonstrated the suitability of this ELISA to detect residues of short-neck clam (*R. philippinarum*) and Sakhalin surf clam (*Pseudocardium sakhalinense*) but did not evaluate it for detection of North American clam species. Because of the sequence identity of this C-terminal peptide across many shellfish species [20], a strong likelihood exists that this ELISA would detect residues of the North American clam species. Our method reported here uses polyclonal antisera capable of detecting multiple clam proteins. The polyclonal diversity may have advantages as various clam proteins could have different fates in response to processing. Our polyclonal antisera were developed against heat-processed clam antigen which favors the likelihood that it would detect processed clam residues, although the ELISA did not work well with detection of retorted clam residues.

Several commercial ELISA kits are marketed for the detection of crustacean tropomyosin residues. In evaluating one of these commercial ELISA kits (Table 4), the kit was able to detect residues from different crustacean shellfish sources (raw and cooked shrimp, lobster, and crab). The theoretical maximal reactivity for shrimp would be 4,800 to 40,320 ppm, based on an average protein content of shrimp of 24% and tropomyosin level of 2 to 16.8% relative to total protein [38]. Thus, the different shellfish species were detected, but not at maximal reactivity. This may be due to variation of tropomyosin across species [38] and to varying immunoreactivity of different types of tropomyosin. This was not further investigated. In contrast to the different shellfish species, clam residues were detected quite weakly with this commercial kit (Table 4). This kit is not suitable for the detection and quantification of traces of clam in other food products.

## 4. Conclusion

Our sandwich ELISA for clam is sensitive and specific and has the potential to provide food industry and regulatory agencies with a useful tool, hitherto unavailable, to control the unintentional presence of clam in food products. Food processing at high temperature limits the reactivity in the ELISA, and analytical data obtained for such processed food samples should be evaluated with care.

## Figures and Tables

**Figure 1:** *Electrophoretic pattern of clam protein extracts and immunoreactivity of clam antisera*. (a) SDS-PAGE with Coomassie staining. (b) Immunoblot with sheep serum. (c) Immunoblot with rabbit serum. Mix (Ret.): mix of Atlantic Surf clam and ocean quahog calm, retorted; Surf: Atlantic Surf clam; Quahog: quahog clam; MWs: molecular weight markers (indicated in kDa at right margin of (a)); +: cooked material; -: raw material. (b) and (c) are aligned with (a) to allow estimating the MWs on the immunoblot, as MW markers do not stain in immunoblot.

**Figure 2:** *Standard curve of the sandwich ELISA for clam protein.* The graph shows the response of various concentrations of clam protein, expressed as parts per million clam protein relative to unextracted sample weight.

**Table 1:** Cross-reactivity of food ingredients of plant and animal origin except seafood.

Tested sample (alphabetic order)	Cross-reactivity (%)	Tested sample (alphabetic order)	Cross-reactivity (%)
Allspice (ground)	<0.02	Peanut flour	<0.02
Barley malt	<0.02	Potatoes (raw)	<0.02
Basil leaves	<0.02	Potato flour	<0.02
Bell pepper (green)	<0.02	Potato starch	<0.02
Bell pepper (red)	<0.02	Refined canola oil	<0.02
Brown sugar (light)	<0.02	Refined corn oil	<0.02
Caramel color	<0.02	Refined peanut oil	<0.02
Carrots (raw)	<0.02	Refined soybean oil	<0.02
Chick pea	<0.02	Refined sunflower oil	<0.02
Coconut	<0.02	Rice flour	<0.02
Corn flour	<0.02	Roasted soybeans	<0.02
Corn starch	<0.02	Rolled whole wheat	<0.02
Corn syrup (light)	<0.02	Romano cheese	<0.02
Corn syrup (high fructose)	<0.02	Salt	<0.02
Cumin (ground)	<0.02	Skim milk powder	<0.02
Egg (whole)	<0.02	Sodium alginate	<0.02
Egg white	<0.02	Soy flour (defatted)	<0.02
Garlic powder	<0.02	Soy isolate	<0.02
Garlic salt	<0.02	Soy lecithin	<0.02
Garlic (minced dried)	<0.02	Soy sauce (acid hydrolyzed)	<0.02
Ginger powder	0.02	Soy sauce (naturally fermented)	<0.02
Guar gum	<0.02	Sugar	<0.02
Honey	<0.02	Thyme	<0.02
Hydrogenated vegetable oil (fully)	<0.02	Tomato paste	<0.02
Hydrogenated vegetable oil (partially)	<0.02	Textured vegetable protein	<0.02
Lemon juice	<0.02	Unrefined olive oil	<0.02
Lime juice	<0.02	Unrefined peanut oil	<0.02
Lemon & pepper	<0.02	Unrefined sesame oil	<0.02
Malt extract	<0.02	Unrefined soybean oil	<0.02
Molasses	<0.02	Unrefined sunflower oil	<0.02
MSG	<0.02	Vinegar (crystal distilled)	<0.02
Mushrooms—portabella	<0.02	Wheat flour	<0.02
Mushrooms—shitake	<0.02	Wheat gluten	<0.02
Mustard (ground)	<0.02	Whey	<0.02
Onion powder	<0.02	White corn meal	<0.02
Oregano	<0.02	White wine	<0.02
Parmesan cheese	<0.02	Whole wheat flour	<0.02
Paprika	<0.02	Yeast—active dry	<0.02
Parsley	<0.02	Yeast—brewers	<0.02
Pepper, black	<0.02	Yellow corn meal	<0.02
Peanut	<0.02		

**Table 2:** Cross-reactivity of seafoods.

Sample	% cross-reactivity
	Relative to clam
Fish and fish products	
Alaska pollock fillet	<0.02
Surimi (Alaskan pollock)	0.09

Molluscs	
Abalone	0.05
Clam juice^∗^	68
Mussels	1.4
Oysters	<0.02
Scallops	0.23
Snails	<0.02
Squid	<0.02

Crustaceans	
Crab	0.04
Crawfish	<0.02
Lobster	<0.02
Shrimp	<0.02

^∗^As this product contains clam, this is “reactivity” rather than “cross-reactivity”.

**Table 3:** Recovery of spikes of clam protein in different model food products.

Spike level (ppm clam protein)	Tomato juice				Potato cream soup				Retorted potato cream soup			
	Sample A (ppm)	Sample B (ppm)	Mean (ppm)	Recovery (%)	Sample A (ppm)	Sample B (ppm)	Mean (ppm)	Recovery (%)	Sample A (ppm)	Sample B (ppm)	Mean (ppm)	Recovery (%)
0	<	<	<	N.A.	<	<	<	N.A.	<	<	<	N.A.
5	<	<	<	N.A.	<	<	<	N.A.	<	<	<	N.A.
10	8.0	6.8	7.4	74	11.2	11.4	11.3	113	<	<	<	N.A.
25	15.5	17.0	16.3	65	24.0	25.5	24.8	99	<	<	<	N.A.
50	33.8	33.6	33.7	67	45.5	43.1	44.3	89	11.6	12.5	12.1	24
100	70.3	66.5	68.4	68	82.5	65.0	73.8	74	29.5	26.3	27.9	28

< Below LLOQ, 6 ppm; N.A.: not applicable. All standards were extracted in duplicate, and each extract was analyzed in triplicate in two different ELISA trials.

**Table 4:** Reactivity of crustacea and clam in the commercial Crustacean Tropomyosin Kit.

Sample	Reactivity
	ppm tropomyosin
Raw shrimp	3389
Cooked shrimp	3716
Lobster	2794
Crab	975
Clams	0.4

## Data Availability

The laboratory data used to support the findings of this study are included within the article.
